The article "Quantitative Analysis of Cone-Beam Computed Tomography Artifacts Induced by Nonmetallic Root Canal Filling Materials Using Different Fields of View: In Vitro Study" was published in 2022. Journal: Scanning.

# Quantitative Analysis of Cone-Beam Computed Tomography Artifacts Induced by Nonmetallic Root Canal Filling Materials Using Different Fields of View: *In Vitro* Study

**DOI:** 10.1155/2022/4829475

**Published:** 2022-02-22

**Authors:** Rahaf A. AlMohareb, Reem M. Barakat, Mohamed Mehanny

**Affiliations:** ^1^Department of Clinical Dental Sciences, College of Dentistry, Princess Nourah bint Abdulrahman University, P.O. Box 84428, Riyadh 11671, Saudi Arabia; ^2^Basic Dental Science, College of Dentistry, Princess Nourah Bint Abdulrahman University, Riyadh, Saudi Arabia

## Abstract

Cone-beam computed tomography (CBCT) imaging artifacts can hinder accurate diagnosis of several conditions. The aim of this study was to quantify CBCT artifacts created by nonmetallic root canal filling materials using two fields of view (FOV). Root canals of twenty extracted maxillary central incisors (*n* = 20) were instrumented and randomly divided into four equal groups: canals in Group 1 were filled with gutta-percha, canals in Group 2 with mineral trioxide aggregate (MTA) and gutta-percha, canals in Group 3 with gutta-percha and glass-fiber posts, and canals in Group 4 with MTA and glass-fiber posts. Each tooth was mounted on a silicon block and scanned three times using a CBCT machine, first with a prefilling scan (control) and then with postfilling scans, using two different FOV (40∗50 mm and 80∗50 mm). Imaging software was used to measure grayscale pixel values of canal cross sections. Data were analyzed using *t*-test and paired *t*-test statistical tests, with statistical significance set at *p* ≤ 0.05. Dentin at the apical and middle third of the teeth showed a significant decrease in minimum grayscale values in association with gutta-percha (*p* = 0.027, *p* = 0.034). However, a wide 80∗50 FOV showed a significant increase in maximum grayscale values of coronal (*p* = 0.048) and apical dentin (*p* = 0.049). Glass-fiber posts in middle third cross sections also corresponded to an increase in maximum grayscale values (*p* = 0.018). Gutta-percha produced dark band artifacts in the root's middle and apical thirds, whereas white streak artifacts were produced by gutta-percha in the coronal third and glass-fiber posts in the coronal and middle thirds when imaged with a wider FOV. A smaller FOV is therefore recommended for CBCT imaging, as it produces fewer artifacts.

## 1. Introduction

Accurate radiographic examination is necessary for successful endodontic diagnosis and treatment preparation, as well as for determining the treatment outcome. Previously, radiographic analysis in endodontics was primarily performed using conventional periapical radiography, which provides a two-dimensional (2D) depiction of three-dimensional (3D) anatomical structures. However, this imaging is plagued with errors due to overlapping structures and the likelihood of distortion [1]. Because of its ability to capture 3D images, cone-beam computed tomography (CBCT) has become an effective imaging modality in dentistry, with proven broad therapeutic and diagnostic capabilities [2]. Many authors advocate CBCT imaging as an additional sensitive and precise diagnostic tool, particularly in endodontic cases [2–4].

Endodontically treated teeth are filled with a number of materials that, due to their composition, create artifacts on CBCT imaging that reduce image quality [5]. Most research has focused on assessing the effect of artifacts from metallic materials (metal posts placed in the root canal) [6–8]. However, the most common root canal filling materials are nonmetallic, most notably gutta-percha, mineral trioxide aggregate (MTA), and, more recently, glass-fiber posts, which have proven to be superior to metal posts in terms of survival rate [9]. Gutta-percha cones are the material of choice for filling the entirety of root canals after endodontic procedures. These cones are made from organic (gutta-percha) and inorganic (zinc oxide and barium sulfate) components [10–12]. MTA is a root filling material widely used in apical surgery, perforation repair, apexification therapy, obturation of open apices, and root resorption due to its high biocompatibility, low solubility, and ability to seal. It is typically confined to filling the section of the root canal in direct contact with periodontal tissue (apical third). It is made of Portland cement, with bismuth oxide added to increase its radio-opacity [13]. Glass-fiber posts are made of a high-mechanical-resistant epoxy resin, which serves as an intracanal dental structure that holds the restoration material in place [14].

CBCT image artifacts may appear as a combination of white streaks and dark bands and are caused by high-density materials [15]. Dark bands may be confused with root fracture in CBCT images [16], which reduces the reliability of CBCT as a diagnostic method. While these artifacts cannot be completely removed, they can be minimized by using lower-density materials, different CBCT imaging settings (such as fields of view (FOV), kVp, mA, and voxel sizes), or by applying artifact reduction algorithms to CBCT images [8].

While many studies explored the artifacts created by metallic root canal filling materials using qualitative and quantitative methods [6, 17, 18], there are limited studies that attempt to quantify artifact production caused by nonmetallic materials, in addition to examine the effect of FOV [14, 19]. Quantitative assessment using mean grayscale pixel value proved to be inaccurate due to different factors such as grayscale nonuniformity, scatter radiation, and beam hardening [18]. Previous studies have proposed using minimum and maximum grayscale values to objectively assess artifact production [20, 21]. Therefore, the purpose of this study was to quantify CBCT artifacts created by different root canal filling materials by measuring the maximum and minimum grayscale pixel values using two different FOV at standard resolution. The rationale of our study has been justified as the artifacts created by discrete materials may not be correctly exhibited depending on multifactorial entities. The null hypothesis was that no significant difference existed between nonmetallic root canal filling materials in creation of CBCT artifacts.

## 2. Materials and Methods

This randomized cross-sectional in vitro study was approved by Princess Nourah Bint Abdulrahman University Institutional Review Board, Riyadh, Saudi Arabia (approval no. 21-0129).

### 2.1. Sample Selection

This study was conducted on twenty extracted human maxillary central incisors (*n* = 20) with comparable diameters that facilitated proportional circular measurements. The selected teeth had been inspected under an operating microscope (A3 series, Global Surgical Corporation, USA) for visible root cracks and fractures. Periapical radiographs were also taken to exclude the presence of root resorption or calcification, more than one root canal, or dilaceration and open apices. The teeth were debrided with ultrasonic scalers and then immersed in saline. During the preliminary CBCT scan, canal and root diameters were measured to exclude oval canals and/or roots. The sample size was calculated using G∗Power 3.1 software, considering a margin of error *α* of 0.05, power (1 − *β*) = 0.95, and an effect size *d* = 1.8. Previous studies that assessed artifacts created by root canal filling materials were conducted on a similar sample size [19, 22–24].

Endodontic access burs were used to prepare access cavities. A size 10 K-file (Dentsply Maillefer, Ballaigues, Switzerland) was used to measure the working length by determining the presence of the file tip at the apical foramen through magnification (X3 dental loupes, JTL, Gobiz, Korea) and subtracting 0.5 mm from that length. Root canal cleaning and shaping for all teeth were performed by one endodontist, using a crown-down technique with ProTaper Universal rotary nickel–titanium files (Dentsply Maillefer, Ballaigues, Switzerland) on a 16 : 1 contra-angle handpiece driven by an electric engine (X-Smart Endodontic Rotary Motor, Dentsply Sirona, United States) at 350 rpm. Preparation was carried out according to the manufacturer's instructions until file F3 with a tip size 30 and variable taper. Throughout preparation, irrigation for every canal was performed using 2 mL of 5.25% NaOCl after each file, followed by 17% EDTA (MD-ChelCream, Meta Biomed, Korea) for 5 minutes to remove the smear layer. The final rinse was performed with 3 mL distilled water, after which the root canals were dried with paper points.

### 2.2. Phantom Preparation

Each tooth was mounted separately on a coded block made from silicon impression putty. The block was immersed in a container filled with water to simulate soft tissues [8, 25, 26]. A circular customized depression was made in the center of the container, into which the tooth model was seated with further adjustment by the light visors of the machine. The individual tooth setup was chosen to quantify the artifacts generated by root canal filling materials, eliminating overlap of artifacts caused by adjacent teeth and/or other tissue. All teeth were scanned after endodontic instrumentation by the same radiologist using a CBCT machine (Planmeca ProMax 3D Mid, Helsinki, Finland). The imaging parameters were set as follows: 12 mA, 90 kVp with FOVs 40∗50 mm and 50∗80 mm. The CBCT data of the selected teeth were reconstructed using Romexis. All scans were viewed on an LCD Dell monitor with a 24-inch screen and 1920 × 1080 high-definition screen resolution. A prefilling scan was used as a control for each tooth. The blocks were then randomly allocated to the four groups described in Figure 1.

### 2.3. Root Canal Filling

Canals in Group 1 were filled with size F3 gutta-percha cones (Dentsply Sirona, United States) and cemented with AH Plus sealer (Dentsply Sirona, United States) using the single cone technique. In Group 2, the canals were filled with MTA (PD white MTA, Switzerland) using the MAP system (Dentsply Maillefer, Ballaigues, Switzerland) and then backfilled with thermoplasticized gutta-percha (SuperEndo *β*, B&L Biotech, United States) and AH Plus sealer. Canals in Group 3 were filled with gutta-percha cones using the same technique applied in Group 1, followed by the removal of the gutta-percha in the coronal and middle thirds using heat (SuperEndo *α*, B&L Biotech, United States). Post space was constructed for a 10 mm long glass-fiber post system (RelyX Fiber Post, 3M ESPE, St. Paul, MN, USA) using the rotary drill burs of the appropriate RelyX fiber post (2# Fiber Post, 3M ESPE, St. Paul, MN, USA). The fiber post had an apical diameter of 0.80 mm and coronal diameter of 1.60 mm. The irrigation solutions for the post space consisted of 5 mL of 2.5% NaOCl, followed by 10 mL of distilled water for 30 seconds. The post space was then dried with absorbent paper points. A try-in was carried out to ensure post fit within the prepared space, followed by cleaning the posts with ethanol. According to the manufacturer's instructions, a self-adhesive resin cement (RelyX Unicem, 3M ESPE, St. Paul, MN, USA) was applied to the root canal using an extension tip. With finger pressure, the fiber posts were promptly placed into the prepared spaces. For 40 seconds, a 1200 mW/cm^2^ LED light curing unit (Elipar S10, 3M ESPE, St. Paul, MN, USA) was used to illuminate the cement and post via the cervical section of the root. Throughout the curing operation, the light curing tip was held near the tooth's surface. Finally, in Group 4, the apical third of the canals was filled with MTA (as in Group 2), followed by glass-fiber postcementation using the same technique as in Group 3.

### 2.4. Image Acquisition and Assessment

After filling the root canals, each tooth was scanned twice: once using an FOV of 40∗50 mm (height∗diameter) cylinder and once using an FOV of 80∗50 mm at 90 kVp and 8 mA with a standard resolution protocol. The FOV protocol (80∗50 mm) enhances acquisition time and therefore generates more images (Figure 2).

The corresponding data set was stored as digital imaging and communications in medicine (DICOM) files with codes corresponding to tooth, root filling materials, and parameter protocol. Planmeca Romexis 6.0 software was used to assess the images.

### 2.5. Objective Analysis via Grayscale Measurements

For pre- and postfilling scans, the entire root length (from the cementoenamel junction to the root apex) was divided into three horizontal segmental lines perpendicular to the longitudinal root axis: a cervical line at 2 mm from the cementoenamel junction, a middle line at the midway point of the entire root length, and an apical line at 2 mm from the apical foramen. Two observers with 10 years of CBCT image analysis expertise analyzed the three axial cross-sectional levels using a standardized region of interest selected for each cross section. Each tooth sample was centralized in FOV during data acquisition. 2D images were exported to ImageJ (version 5.2, LOCI, University of Wisconsin), where the canal content in pre- and postfilling scans was defined and deducted from the images using the threshold function. Grayscale pixel values in the dentine canal cross sections were then measured and recorded. A decrease in minimum grayscale values between pre- and postfilling images would indicate the presence of hypodense (dark) artifacts, whereas an increase in maximum grayscale values would be associated with hyperdense (white streak) artifacts. Measurements were repeated after a period of 3 weeks to increase the reliability of results.

### 2.6. Statistical Analysis

The data were analyzed using SPSS version 22 (IBM Corp., USA). Normality of the data was explored using the Shapiro–Wilk test. Accordingly, data were compared using the *t*-test and paired sample *t*-test after grouping canal filling materials into two groups: gutta-percha and glass-fiber post for coronal third and middle third cross sections and gutta-percha and MTA for apical third cross sections. Inter- and intrarater reliability was tested using the 95% confidence interval interclass correlation coefficient (ICC). The significance level was set at a *p* value of <0.05.

## 3. Results

### 3.1. Inter- and Intrarater Reliability for Grayscale Values

The ICC showed that both inter and intrarater reliability ranged from 0.990 to 1.000, indicating excellent to perfect agreement.

### 3.2. Comparison between Radiodensity of Obturation Materials

#### 3.2.1. Coronal and Middle Third Cross Sections

Glass-fiber posts resulted in lower maximum values when compared with gutta-percha, but a significant difference was found only for values in the middle third cross sections taken at 80∗50 FOV (*p* = 0.027).

#### 3.2.2. Apical Third Cross Sections

The maximum values recorded for MTA were significantly lower compared with those for gutta-percha in both FOV (*p* = 0.010 and *p* ≤ 0.001).

### 3.3. Comparison between Grayscale Values of Canal Cross Sections

Pairing the pre- and postobturation scans revealed that gutta-percha was associated with a significant decrease in minimum grayscale values, which corresponds to the formation of hypodense (dark) artifacts in the middle third cross sections, regardless of the FOV used (*p* = 0.027, *p* = 0.034). This also occurred in the apical third when the small 40∗50 FOV was used (*p* = 0.005) (Table 1). MTA, however, was not associated with any significant changes in grayscale values (Table 2).

In the coronal third, regardless of FOV, gutta-percha was associated with a significant shift in the grayscale values in the dentine cross section toward values that were less negative, indicating hyperdense changes (*p* = 0.001, *p* ≤ 0.001) (Table 1). When imaged with an 80∗50 wide FOV, there was also a significant increase in maximum grayscale values (corresponding to hyperdense artifacts in canals obturated with gutta-percha in the coronal (*p* = 0.048) and apical (*p* = 0.049) thirds, as well as in the middle third of canals obturated with glass-fiber posts (*p* = 0.018)) (Tables 1 and 2).

No significant differences were found in comparison of the maximum and minimum grayscale values of coronal or middle third cross sections filled with gutta-percha or glass-fiber posts, regardless of FOV (Table 3).

## 4. Discussion

The long-term success of endodontic treatment is determined by a variety of criteria, including the quality of endodontic therapy, retained tooth structure, and selection of the appropriate filling material. The composition of this filling material often produces artifacts in CBCT images that reduce image quality [5] and can hinder accurate diagnosis of certain conditions, such as root fracture [16]. The effect of filling materials on CBCT images has been widely studied [25, 27–31]. The novelty of the present study is that it addresses the quantification (objective assessments) of CBCT artifacts by measuring the pixel values of different nonmetallic root canal filling materials using two different FOV.

A previous study by Brito-Júnior et al. [29] counted the amount of white streak artifacts produced using CBCT. Their method of analyzing artifacts, however, was plagued by several issues affecting the reliability of their results. These issues included the inability to differentiate the direction of the streaks created by various materials, the nonuniformity of the teeth studied, and the transmission of white streak or dark band artifacts created by adjoining teeth. In this study, teeth were scanned separately to avoid such interferences. Many studies have advocated using grayscale values to quantify CBCT artifacts [17, 21]. In order to assess grayscale variations between the gutta-percha, glass-fiber post, and MTA groups, an objective analysis of the maximum and minimum grayscale values was performed for each group. Grayscale analysis was performed individually for each tooth cross section and material, in order to quantify the artifacts generated by these root canal filling materials. This is consistent with Smeets et al. [32], who reported a discrepancy in the distribution of grayscale values in a CBCT image when compared with reference values. This would result in distinct images that reflect the effect of the different materials.

There is a positive association between the mineral content of a material and CBCT image artifacts; the higher the mineral content, the greater the number of artifacts [17, 21, 33]. The results of this study showed that the radiodensity of gutta-percha in the apical third had significantly higher maximum grayscale values than MTA and glass-fiber posts in the coronal and middle thirds of the root. This discrepancy in the maximum grayscale values could be explained by the high content of inorganic components (such as zinc oxide and barium sulfate) in their composition, as well as the AH Plus sealer material used to cement the gutta-percha cones in the canal [23].

Comparison of the grayscale values of the tooth cross sections in scans before and after obturation revealed that the use of gutta-percha with the AH Plus sealer resulted in significantly higher maximum values in the coronal (80∗50 FOV) and apical thirds (40∗50 FOV). This is in agreement with Salineiro et al. [21], who found a higher number of white streak artifacts (maximum grayscale values) in coronal root thirds filled with gutta-percha. Moreover, the glass-fiber posts produced significantly higher maximum values in the coronal and middle third at 80∗50 FOV, whereas the MTA did not have statistically significant maximum grayscale values in the apical third at either FOV. This is likely because white MTA (used here) produces fewer artifacts than gray MTA, due to the lack of iron in its composition [23].

Previous studies have suggested that the higher number of white artifacts in coronal sections was due to the scattering effect created by root canal filling materials or metal restorations in the image, which produced a high linear density (bright lines) [21, 34]. Samples in this study were therefore analyzed without crown restorations to avoid scattering artifacts and measure the maximum grayscale values of the filling materials individually. Measuring the maximum pixel values of the filling materials used yielded a higher maximum value for gutta-percha compared with glass-fiber posts and MTA. This is consistent with the findings of Fox et al. [35], who reported that gutta-percha, a distinctly visible material on conventional intraoral images, produced significant artifacts that affected CBCT image quality. This is due to its radiopaque properties related to the proportions of inorganic filler, which contains zinc and barium.

In endodontically treated teeth, the coronal and middle root thirds suffer considerable structural loss and, as a result, experience the highest frequency of root fractures [36]. In these areas, accurate image interpretation is therefore critical to distinguish between artifacts caused by canal filling materials and root fracture, particularly when the patient presents with symptoms consistent with the latter. The results of this study showed that gutta-percha produced significantly higher percentage minimum values (dark areas that could mimic a root fracture) in the middle third at both FOVs and in the apical third at 40∗50 FOV. This is consistent with Andreasen et al. [37], who reported that the middle third of the root was the area with the greatest grayscale variation, and with Salineiro et al. [21], who found a greater number of dark bands in the coronal and middle third of the root. Both of these areas are therefore at greater risk of root fracture misdiagnoses.

In this study, the ICC showed excellent inter- and intrarater agreement, supporting the reproducibility of the chosen methodology and grayscale analysis. As this in vitro study did not imitate the complex layout of teeth in the oral cavity, the findings presented above may not be directly applicable clinically. Nevertheless, the results do suggest that FOV has an effect on final image quality, depending on the type of root canal filling material used. In root canals filled using glass-fiber posts, increasing the FOV resulted in a statistically significant increase in white streak artifacts in the coronal and middle root planes. This also proved to be the case in the coronal third when gutta-percha was used as filling. From these findings, we conclude that a smaller FOV with a standard resolution protocol is preferable to minimize artifact production and patient dose.

Another factor that contributes to artifact formation is the thickness of individual teeth, which can result in different attenuation values, despite uniform canal instrumentation. The distribution pattern of artifacts in tomographic imaging is multifactorial. In our study, there was a significant positive correlation when the wider FOV (80∗50) was used. When a small FOV was used, only the minimum values recorded in the middle third were positively associated with the tooth surface in the area. Thus, the interaction between beam hardening and scattering can lead to variations in the distribution of artifacts in CBCT images.

## 5. Conclusions

Objective analysis of root canal filling materials showed that gutta-percha had higher grayscale values than glass-fiber posts and MTA when imaged using CBCT. Gutta-percha produced significantly greater dark band artifacts in the middle and apical third of the root, which may compromise accurate diagnosis of root fracture and lead to poorer prognosis for the tooth. In contrast, a wider FOV produced significantly greater white streak artifacts in the coronal third when using gutta-percha and in the coronal and middle third when using glass-fiber posts. A smaller FOV is therefore highly recommended for CBCT imaging, as it produces fewer artifacts.

## Figures and Tables

**Figure 1:** Methodology flowchart.

**Figure 2:** Samples of middle and apical third CBCT images using both fields of view.

**Table 1:** Paired *t*-test for pre- and postobturation scans in the coronal and middle thirds.

Section	Material	FOV	Value	Mean	Std. dev.	Std. error	95% confidence interval of the difference		*t*	df	Sig.
							Lower	Upper			
Coronal third	Gutta-percha	40∗50	Min	8.200	28.642	9.057	-12.289	28.689	0.905	9	0.389
			Max	-2.200	4.211	1.331	-5.212	0.812	-1.652	9	0.133
			Skew.	-0.774	0.497	0.157	-1.130	-0.418	-4.921	9	0.001^∗^
		80∗50	Min	-0.300	35.882	11.347	-25.968	25.368	-0.026	9	0.979
			Max	3.900	5.384	1.702	0.0484	7.751	2.291	9	0.048^∗^
			Skew.	1.038	0.582	0.184	0.621	1.454	5.638	9	0.000^∗^
	Glass-fiber post	40∗50	Min	-2.900	32.925	10.412	-26.453	20.653	-0.279	9	0.787
			Max	-1.800	3.735	1.181	-4.472	0.872	-1.524	9	0.162
			Skew.	-0.478	0.914	0.289	-1.132	0.175	-1.656	9	0.132
		80∗50	Min	7.100	26.768	8.464	-12.048	26.248	0.839	9	0.423
			Max	1.700	1.828	0.578	0.391	3.008	2.940	9	0.016^∗^
			Skew.	0.406	0.703	0.222	-0.097	0.909	1.825	9	0.101

Middle third	Gutta-percha	40∗50	Min	12.800	15.310	4.841	1.847	23.752	2.644	9	0.027^∗^
			Max	-4.400	6.203	1.961	-8.838	0.0380	-2.243	9	0.052
			Skew.	-0.0743	0.556	0.175	-0.472	0.323	-0.422	9	0.683
		80∗50	Min	-19.400	24.495	7.746	-36.923	-1.876	-2.504	9	0.034^∗^
			Max	2.000	5.477	1.732	-1.918	5.918	1.155	9	0.278
			Skew.	-0.025	0.633	0.200	-0.478	0.427	-0.126	9	0.903
	Glass-fiber post	40∗50	Min	-3.500	26.437	8.360	-22.412	15.412	-0.419	9	0.685
			Max	-2.500	4.453	1.408	-5.685	0.685	-1.775	9	0.110
			Skew.	0.040	0.434	0.137	-0.270	0.351	0.295	9	0.775
		80∗50	Min	3.400	22.652	7.163	-12.804	19.604	0.475	9	0.646
			Max	4.500	4.904	1.551	0.991	8.008	2.901	9	0.018^∗^
			Skew.	0.097	0.515	0.163	-0.271	0.466	0.599	9	0.564

^∗^ *p* ≤ 0.05.

**Table 2:** Paired *t*-test for pre- and postobturation scans in the apical third.

Material	FOV	Value	Mean	Std. dev.	Std. error	95% confidence interval of the difference		*t*	df	Sig.
						Lower	Upper			
Gutta-percha	40∗50	Min	23.700	20.066	6.345	9.345	38.054	3.735	9	0.005^∗^
		Max	-3.400	6.16	1.950	-7.812	1.012	-1.743	9	0.115
		Skew.	0.284	1.457	0.461	-0.758	1.326	0.616	9	0.553
	80∗50	Min	12.300	28.158	8.904	-7.843	32.443	1.381	9	0.201
		Max	5.700	7.931	2.508	0.0265	11.373	2.273	9	0.049^∗^
		Skew.	-0.114	1.297	0.410	-1.043	0.813	-0.280	9	0.786

MTA	40∗50	Min	-4.500	25.526	8.072	-22.760	13.760	-0.557	9	0.591
		Max	-1.000	8.055	2.547	-6.762	4.762	-0.393	9	0.704
		Skew.	0.270	0.814	0.257	-0.312	0.852	1.049	9	0.321
	80∗50	Min	1.000	28.087	8.881	-19.092	21.092	0.113	9	0.913
		Max	0.000	8.666	2.740	-6.199	6.199	0.000	9	1.000
		Skew.	-0.442	0.678	0.214	-0.927	0.042	-2.063	9	0.069

^∗^ *p* ≤ 0.05.

**Table 3:** Comparing minimum and maximum grayscale values for gutta-percha and glass-fiber posts.

FOV	Section level	Grayscale values	Material	*N*	Mean	Std. error	Sig.
4∗5	Coronal third	Min	Gutta-percha	10	153.200	11.0653	0.184
			Glass-fiber post	10	171.100	6.7486	
		Max	Gutta-percha	10	251.900	1.9117	0.436
			Glass-fiber post	10	253.500	0.6191	
	Middle third	Min	Gutta-percha	10	169.100	4.8108	0.506
			Glass-fiber post	10	174.300	5.9648	
		Max	Gutta-percha	10	251.100	1.1590	0.212
			Glass-fiber post	10	248.700	1.4457	

8∗5	Coronal third	Min	Gutta-percha	10	161.100	11.7260	0.319
			Glass-fiber post	10	175.300	7.3591	
		Max	Gutta-percha	10	253.600	0.7775	0.844
			Glass-fiber post	10	253.400	0.6360	
	Middle third	Min	Gutta-percha	10	162.500	7.1184	0.293
			Glass-fiber post	10	174.200	8.1128	
		Max	Gutta-percha	10	248.700	1.0333	0.177
			Glass-fiber post	10	250.700	0.9781	

^∗^ *p* ≤ 0.05.

## Data Availability

The data that support the findings of this study are available on request from the corresponding author.
